RETRACTED

# Evaluation of the Effectiveness of Artificial Intelligence Chest CT Lung Nodule Detection Based on Deep Learning

**DOI:** 10.1155/2021/9971325

**Published:** 2021-08-17

**Authors:** Fukui Liang, Caiqin Li, Xiaoqin Fu

**Affiliations:** Changle People Hospital, Weifang 262400, Shandong, China

## Abstract

Lung cancer is one of the most malignant tumors. If it can be detected early and treated actively, it can effectively improve a patient's survival rate. Therefore, early diagnosis of lung cancer is very important. Early-stage lung cancer usually appears as a solitary lung nodule on medical imaging. It usually appears as a round or nearly round dense shadow in the chest radiograph. It is difficult to distinguish lung nodules and lung soft tissues with the naked eye. Therefore, this article proposes a deep learning-based artificial intelligence chest CT lung nodule detection performance evaluation study, aiming to evaluate the value of chest CT imaging technology in the detection of noncalcified nodules and provide help for the detection and treatment of lung cancer. In this article, the Lung Medical Imaging Database Consortium (LIDC) was selected to obtain 536 usable cases based on inclusion criteria; 80 cases were selected for examination, artificial intelligence software, radiologists, and thoracic imaging specialists. Using 80 pulmonary nodules detection in each case, the pathological type of pulmonary nodules, nonlime tuberculous test results, detection sensitivity, false negative rate, false positive rate, and CT findings were individually analyzed, and the detection efficiency software of artificial intelligence was evaluated. Experiments have proved that the sensitivity of artificial intelligence software to detect noncalcified nodules in the pleural, peripheral, central, and hilar areas is higher than that of radiologists, indicating that the method proposed in this article has achieved good detection results. It has a better nodule detection sensitivity than a radiologist, reducing the complexity of the detection process.

## 1. Introduction

With the progress of human society, the development of science and technology, and the improvement of people's living standards, health issues have become the focus of attention. Because of its high incidence, high mortality, low cure rate, and low survival rate, lung cancer is a malignant tumor with high mortality, making it the number one killer that threatens human survival and affects the quality of human life. The initial symptom of lung cancer is a lung nodule. The irregular shape, large gray range change, and variable scale complicate the image manifestation of pulmonary nodules, leading more researchers to evaluate the effectiveness of pulmonary nodule detection.

RETRACTED

With the development of medical imaging technology, CT imaging has gradually become one of the most popular imaging methods for diagnosing diseases. Currently, thin-slice spiral chest CT imaging has achieved submillimeter resolution and has high sensitivity in finding small and hidden nodules. However, due to the large number of slices in CT images and the abundant blood vessels and airway structures in the lungs, the diagnosis becomes more complicated and the false positive rate is also higher. Due to the disadvantages of traditional artificial chest imaging in the diagnosis of chest diseases, such as heavy workload, long reading cycle, and strong subjectivity, a fast, accurate, and reproducible artificial intelligence chest CT detection system for lung nodules is required to assist doctors in diagnosing diseases.

Early detection of lung cancer in Ma et al. via low-dose computed tomography (LDCT) may reduce mortality. However, LDCT increased the number of uncertain pulmonary nodules (PNs), and 95% of PNs eventually turned out to be false positives. There is an urgent need for a method specifically used to differentiate between malignant and benign PNs. They previously identified a set of peripheral blood mononuclear cell (PBMC) miRNA (miRs-19b-3p and -29b-3p) biomarkers for lung cancer. This study aims to evaluate the effectiveness of integrated biomarkers and the clinical and radiological characteristics of smokers to distinguish between malignant and benign PN. The expression of PBMC in the training set of 137 individuals with PN was analyzed. Use multiple logistic regression analysis to develop predictive models based on biomarkers, radiological characteristics of PNs, and clinical characteristics of smokers to identify malignant PNs. The performance of the predictive model was verified on a test set of 111 subjects using PN. A predictive model containing two biomarkers (PNs and the exact location of the smoking year) was set up and the area under the model curve was 0.91. Their experiment constituted a predictive model, but they did not test the control variable factors, so they need to see the experimental data reasonably [1]. Hassabis et al. neuroscience and artificial intelligence (AI) have a long and intertwined history. However, in the recent era, communication and collaboration between these two fields have become less common. As a summary, they focused on sharing topics, which may be the key to promoting future research in these two fields. However, artificial intelligence can also be applied to a variety of different fields, and they did not conduct a deeper research [2]. The purpose of the Nguyen et al. study is to measure the prevalence of lung cancer screening for clinically significant extrapulmonary findings on chest CT in the National Lung Screening Test (NLST) in the United States. For a retrospective analysis of the extrapulmonary findings of 17,309 participants who underwent low-dose screening chest CT during the NLST period from August 2002 to September 2007, readers of NLST radiologists code these findings as “minor” or “potentially significant.” Based on the written description of the review records, the results of extrapulmonary examinations were divided into five organ groups (cardiovascular, thyroid, adrenal, kidney, liver, and gallbladder). The extrapulmonary malignancies diagnosed during the screening were also identified from the medical and vital status records of the same population. The prevalence of organ-specific findings and newly diagnosed extrapulmonary malignancies was calculated. An exemption from the review of human subjects was received. 58.7% of CT screening participants noticed extrapulmonary findings, while 19.6% of the findings were coded as potentially important. But they still need to conduct more experiments to prove the accuracy of the results [3].

RETRACTED

The research in this article is mainly based on deep learning-based artificial intelligence chest CT lung nodule detection efficiency evaluation. The structure of the article is mainly from the introduction to the introduction of the research methods in this article to the design of chest CT lung nodule detection experiments and finally the detection results performance analysis. The innovation of this paper is that, based on the rationale of deep learning and artificial intelligence, there is an innovative research method for pulmonary nodule detection in combination with chest CT technology, so that the detection efficiency evaluation results can be obtained.

## 2. Evaluation of the Effectiveness of Artificial Intelligence Chest CT Pulmonary Nodule Detection

### 2.1. Deep Learning

In deep learning, by studying the inherent laws and representation levels of massive data samples, the simple features at the bottom are combined to form more abstract high-level composite features, and the distributed representation of data features is realized. It has become an important part of deep learning algorithms driven by the wave of artificial intelligence [4, 5]. Deep learning is the process of learning a function. The principle is to describe the characteristics of the model and fine-tune the test data by learning the intrinsic characteristics of the original data and the level of abstraction [6].

#### 2.1.1. Deep Learning Framework

With the rapid development of deep learning technology, researchers are no longer satisfied with basic theoretical analysis, and the requirements for practical applications are increasingly being placed. The idea of creating a large-scale deep learning framework is being proposed. The in-depth learning framework can contain basic algorithm modules and provide a solid foundation for the subsequent rapid construction of required models or training, coordination, testing, and development of existing models [7, 8].

RETRACTED

#### 2.1.2. Deep Learning Model

There are connections between neurons in the upper and lower layers of the DBN neural network structure, but there is no connection between neurons in the same layer. The neural unit in the optical layer is mainly used to receive input, and the neural unit in the hidden layer is mainly used to capture the high-order data correlation displayed in the optical layer [9, 10]. Convolutional neural network is a feedforward neural network that uses convolution kernel operations instead of general matrix multiplication operations [11, 12]. Because of the progressive characteristics of its network structure, the extraction of image features is also from low-level simple texture features to high-level complex structure features which gradually change; the final combination is a feature map. Image features extracted based on this representation learning method often have good stability, so convolutional neural networks have huge advantages in processing two-dimensional image data [13, 14].

### 2.2. Lung CT Image and Lung Nodule Detection

#### 2.2.1. CT Imaging Signs of Lung Nodules

1. The growth position of lung nodules and the relationship with surrounding tissues: nodules that are located in the lung parenchyma and do not stick to other tissues and have a clearer boundary are called single lung nodules. Nodules attached to blood vessels are called vascular-adherent pulmonary nodules. It is firmly attached to the pleura or nodule located near the pleura and associated with the pleura and is called a pleural adhesion pulmonary nodule [15, 16]. Compared to detached nodules, adhesive nodules are more likely to be missing or misdetected.
2. External morphology of lung nodules: mainly the shape and edge information of the nodule are considered. Because the lung tumors grow at different speeds in all directions and are blocked by the surrounding tissues, the surface of the tumor will form an arc-shaped concave-convex phenomenon called lobular sign. In addition, the rough edge of the tumor caused by the infiltration and interstitial reaction around the tumor is called burr sign [17, 18]. The thick and blunt structure between the lobular sign and the burr sign is called spinous protrusion. Generally, benign nodules have smooth edges without obvious lobes or burrs, and malignant nodules have irregular edges and protrusions and burrs. Due to differences in the growth position, growth rate, or the influence of surrounding tissues on the nodules, the shape of the nodules is round, semicircular, or other irregular shapes [19].
3. Density of lung nodules: mainly the internal tissue characteristics of lung nodules are investigated. Generally, the density of benign nodules is relatively uniform, while malignant nodules will show cell necrosis and liquefaction as the tumor grows, and even bubbles and voids will form inside, which leads to the uneven density of lung nodules [20]. The CT value of the calcified structure is greater than 100HU. According to the different density of nodules, nodules can be divided into solid, partially solid, or nonsolid lung nodules.

RETRACTED

#### 2.2.2. The Role of CT in Lung Cancer Detection

With the rapid development of CT technology, the acquired CT images are clearer and have higher resolution. CT can play an increasingly important role in the early detection, localization, and lesion characterization of lung cancer and has become a clinical early detection of lung cancer and the most commonly used and most effective method [21–23]. CT images can clearly show the edge, shape, and density of lung nodules and the relationship with adjacent tissues. It can also accurately show the location of hilar and mediastinal lymphatic enlargement, which plays a very important role in determining the stage of lung cancer.

### 2.3. Medical Image Enhancement Algorithm

#### 2.3.1. Image Sharpening Enhancement

*(1) Gradient Operator*. If *f*(*x*, *y*) is the original image, then the gradient value definition formula of *f*(*x*, *y*) at point (*x*, *y*) is expressed as

(1) $$\begin{array}{c} G\left[f\left(x,y\right)\right]=\left[\begin{array}{c} \frac{\partial f}{\partial x}\\ \frac{\partial f}{\partial y} \end{array}\right]. \end{array}$$

The expression of the magnitude of the gradient is as follows:

(2) $$\begin{array}{c} \left|G\left[f\left(x,y\right)\right]\right|=\sqrt{{\left(\frac{\partial f}{\partial x}\right)}^{2}+{\left(\frac{\partial f}{\partial y}\right)}^{2}}. \end{array}$$

Use the lookup operation to approximate equation (3), as shown in the following:

(3) $$\begin{array}{c} \left|G\left[f\left(x,y\right)\right]\right|={\left\{{\left[f\left(x,y\right)-f\left(x+1,y\right)\right]}^{2}+{\left[f\left(x,y\right)-f\left(x,y+1\right)\right]}^{2}\right\}}^{1/2}, \end{array}$$

(4) $$\begin{array}{c} \left|G\left[f\left(x,y\right)\right]\right|\approx \left|f\left(x,y\right)-f\left(x+1,y\right)\right|+\left|f\left(x,y\right)-f\left(x,y+1\right)\right|. \end{array}$$

The size of the gray scale is proportional to the difference between the gray values of adjacent pixels in the two directions. The formula is as follows:

(5) $$\begin{array}{c} g\left(x,y\right)=G\left[f\left(x,y\right)\right],\\ g\left(x,y\right)=\left\{\begin{array}{cc} G\left[f\left(x,y\right)\right], & G\left[f\left(x,y\right)\right]\geq T,\\ f\left(x,y\right), & G\left[f\left(x,y\right)\right]<T. \end{array}\right. \end{array}$$

*T* represents the set threshold value. When the gradient value of a certain area in the image is greater than the threshold value, the pixel gray value of the original image is replaced with the gradient value [24].

*(2) Laplacian.f*(*x*, *y*) represents the image to be enhanced, and the Laplacian differential definition of *f*(*x*, *y*) at point (*x*, *y*) is expressed as follows:

(6) $$\begin{array}{c} \nabla^{2}f\left(x,y\right)=\frac{\partial^{2}f}{\partial x^{2}}+\frac{\partial^{2}f}{\partial y^{2}}, \end{array}$$

and the general expression for enhancement using Laplace is as follows:

(7) $$\begin{array}{c} g\left(x,y\right)=f\left(x,y\right)-A\cdot \nabla^{2}f\left(x,y\right),\\ \nabla^{2}f\left(x,y\right)=\left[f\left(x+1,y\right)+f\left(x-1,y\right)+f\left(x,y+1\right)+f\left(x,y-1\right)\right]-4f\left(x,y\right). \end{array}$$

Since the Laplacian second-order operator can detect a single line segment and a single point in an image, even when the image is affected by noise, even if the bright spot in the dark area becomes brighter, the algorithm will make the noise more influential. Therefore, the antinoise ability of the algorithm must be considered when using the Laplacian operator [25, 26].

RETRACTED

### 2.4. Candidate Lung Nodule Detection

Image preprocessing includes rib removal and lung segmentation. The next step is to screen for suspected lung nodules in the segmented lung area. There are many classical detection methods for suspected lung areas such as difference image technique, multiscale detection, convergence exponent, Hough transform, multiple threshold segmentation, and other methods [27, 28]. Here, the generalized LoG filter kernel spot detection method is used to extract the suspected lung nodules. The definition of Gaussian kernel is given as follows:

(8) $$\begin{array}{c} G\left(x,y,\sigma \right)=\frac{1}{2\pi \sigma^{2}}e^{-\left(\left(x^{2}+y^{2}\right)/2\sigma^{2}\right)}, \end{array}$$

where *σ* is the standard deviation. The Gaussian convolution of image *I*(*x*, *y*) is expressed as

(9) $$\begin{array}{c} L\left(x,y,\sigma \right)=G\left(x,y,\sigma \right)*I\left(x,y\right), \end{array}$$

where *∗* is the convolution operator. The definition of Laplacian is given as follows:

(10) $$\begin{array}{c} \nabla^{2}=\frac{\partial^{2}f}{\partial x^{2}}+\frac{\partial^{2}f}{\partial y^{2}}. \end{array}$$

Then the Laplacian of Gaussian can be expressed as

(11) $$\begin{array}{c} \text{LoG}=\Delta G\left(x,y,\sigma \right)\\ =\frac{\partial^{2}G\left(x,y,\sigma \right)}{\partial x^{2}}+\frac{\partial^{2}G\left(x,y,\sigma \right)}{\partial y^{2}}\\ =\frac{x^{2}+y^{2}+2\sigma^{2}}{2\pi \sigma^{6}}e^{\left(\left(-x^{2}-y^{2}\right)/2\sigma^{2}\right)}. \end{array}$$

If we let Δ*G*(*x*, *y*, *σ*)=0, we can get

(12) $$\begin{array}{c} x^{2}+y^{2}=2\sigma^{2}. \end{array}$$

This shows that the extreme point of the Laplacian of Gaussian satisfies the radius of $\sqrt{2}\sigma$ circle. Since the differential and integral of equation (14) are interchangeable, then,

(13) $$\begin{array}{c} \frac{\text{d}}{\text{d}t}\left[h\left(t\right)*I\left(x,y\right)\right]=\frac{\text{d}}{\text{d}t}\int I\left(\tau \right)h\left(t-\tau \right)\text{d}\tau \\ =\int I\left(\tau \right)\frac{\text{d}}{\text{d}t}h\left(t-\tau \right)\text{d}\tau \\ =I\left(t\right)*\frac{\text{d}}{\text{d}t}h\left(t\right). \end{array}$$

Then, the Laplacian of Gaussian transformation of image *I*(*x*, *y*) is

(14) $$\begin{array}{c} \nabla^{2}\left[G\left(x,y,\sigma \right)*I\left(x,y\right)\right]=\nabla^{2}\left[G\left(x,y,\sigma \right)\right]*I\left(x,y\right)\\ =\Delta G\left(x,y,\sigma \right)*I\left(x,y\right). \end{array}$$

The generalized Gaussian kernel definition is given as follows:

(15) $$\begin{array}{c} G\left(x,y,\sigma_{x},\sigma_{y},\mu_{x},\mu_{y}\right)=\frac{1}{2\pi \sigma_{x}\sigma_{y}}e^{\left(-{\left(x-\mu_{x}\right)}^{2}/2\sigma_{x}^{2}\right)+\left(-{\left(y-\mu_{y}\right)}^{2}/2\sigma_{y}^{2}\right)}, \end{array}$$

where *σ*_*x*_, *σ*_*y*_, *μ*_*x*_, *μ*_*y*_ are the variance and mean, respectively. If we let *σ*=*σ*_*x*_=*σ*_*y*_ and *μ*_*x*_=*μ*_*y*_=0, we have

(16) $$\begin{array}{c} G\left(x,y,\sigma_{x},\sigma_{y},\mu_{x},\mu_{y}\right)=G\left(x,y,\sigma \right)\\ =\frac{1}{2\pi \sigma^{2}}e^{\left(-x^{2}-y^{2}/2\sigma^{2}\right)}. \end{array}$$

At this time, the generalized Gaussian kernel degenerates into a general Gaussian kernel form. When *σ*_*x*_ ≠ *σ*_*y*_ or *μ*_*x*_ ≠ *μ*_*y*_ ≠ 0, the generalized Laplacian Gauss kernel can be expressed as

(17) $$\begin{array}{c} \nabla^{2}\left[G\left(x,y,\sigma_{x},\sigma_{y},\mu_{x},\mu_{y}\right)*I\left(x,y\right)\right]=\nabla^{2}\left[G\left(x,y,\sigma_{x},\sigma_{y},\mu_{x},\mu_{y}\right)\right]*I\left(x,y\right)\\ =\Delta G\left(x,y,\sigma_{x},\sigma_{y},\mu_{x},\mu_{y},\sigma \right)*I\left(x,y\right). \end{array}$$

RETRACTED

## 3. Experimental Design of Artificial Intelligence Chest CT Pulmonary Nodule Detection Efficiency Evaluation

### 3.1. Test Subject

The database selected for this experiment is LIDC, which contains chest CT images of lung cancer patients with diagnostic information, as well as annotation information for pathological images. This data set contains 1018 cases. Each case includes a chest CT image scanned by a hospital and an XML file that records diagnostic information of experienced radiologists. According to the inclusion criteria, 536 usable cases were obtained. Finally, SPSS17.0 software was used for stacking sampling. 80 cases were selected as test objects. The basic characteristics of nodules in 80 cases are shown in Table 1. Using artificial intelligence software, radiologists, and chest imaging experts to refer to intelligent software for lung nodules detection in these 80 cases, respectively, the detection results of pathological types, noncalcified nodules, detection sensitivity, false negative rate, and false positive analyze the CT performance of lung nodules and evaluate the detection efficiency of artificial intelligence software.

Inclusion criteria: there is no problem with the XML file; there is at least one noncalcified nodule; there is a thin-slice chest CT image (thickness = 1.25 mm).

### 3.2. Experimental Method

For each patient's CT picture, select a more appropriate range for observing the lungs and map it to the [0, 255] grayscale interval. The accuracy of each patient's CT scanning machine mainly varies from about 2 mm to 5 mm. The natural image is 3 channels and the CT scan image is single channel. Here, three adjacent slices are selected and combined into one image. The training data selects data from 200 patients as a training set and validation set for training.

### 3.3. Establishment of the Model Evaluation Index System

The evaluation index is a specific evaluation item that is determined according to the evaluation purpose and can reflect the basic characteristics of the evaluation target. Indicators are specific and measurable and are the observation points of your target. Clear conclusions can be drawn from the actual observation of the object. Typically, the metrics system includes three levels of metrics. This is the relationship between gradual decomposition and improvement. Among these, the first-stage evaluation index and the second-stage evaluation index are relatively abstract and cannot be used as direct evaluation criteria. The three-level assessment indicator should be specific, measurable, and action-oriented and can be used as a direct basis for assessment.

### 3.4. Statistical Processing

SPSS23.0 software was used for data processing, and the count data was expressed as a percentage (%), *k* is the number of data in this experiment, *σ*^2^ is the variance of all survey results, and *P* < 0.05 indicates that the difference is statistically significant. The formula for calculating reliability is shown in the following equation:

(18) $$\begin{array}{c} a=\frac{k}{k-1}\left(1-\frac{\sum \sigma_{i}^{2}}{\sigma^{2}}\right). \end{array}$$

RETRACTED

## 4. Artificial Intelligence Chest CT Pulmonary Nodule Detection Efficiency Evaluation

### 4.1. Evaluation Index System Based on Index Reliability Testing

Here we perform reliability analysis on all reliability indicators of each object, and the reliability indicators we choose for each object are slightly different. The results are shown in Table 2.

It can be seen from Figure 1 that the pathological type detection results, the detection results of noncalcified nodules, and the detection results and the data obtained from the CT manifestations of lung nodules have a very good effect on this experiment (*α* > 0.8); the data obtained from the false negative rate of lung nodule detection and the false positive rate of lung nodule detection have an acceptable impact on this experiment (*α* > 0.7), indicating that in this article that is studying surgery the six indicators selected for the prevention of gastrointestinal surgical incision infection are reasonable in laboratory nursing intervention, which provides a basis for the follow-up experiments.

### 4.2. Evaluation of Lung Nodule Detection Efficiency

#### 4.2.1. Pathological Type Detection Results

Here we analyze the results of lung nodule detection in these 80 cases based on artificial intelligence software, radiologists, and chest imaging experts with reference to intelligent software. The results are shown in Table 3.

It can be seen from Table 3 that there are a total of 59 benign nodules and 21 malignant nodules in 80 patients with lung nodules, which can all be detected by artificial intelligence software, radiologists, and chest imaging experts with reference to intelligent software.

#### 4.2.2. Analysis Based on Detection Sensitivity

Here we use artificial intelligence software and radiologists to determine the authenticity of the nodules and use the chest imaging expert to refer to the intelligent software to detect the authenticity of the nodules. The result is the total number of true nodules. The results are shown in Table 4.

In Table 4 and Figure 2, as a result of checking the authenticity of nodules by a chest imaging expert referring to intelligent software, 236 real nodules were finally determined, and a total of 234 true nodules were determined by artificial intelligence software; the sensitivity is 99.15%; the radiologist detected 112 real nodules and the sensitivity was 47.45%. The sensitivity of artificial intelligence software to detect uncalcified nodules was significantly higher than that of radiologists, and the difference was statistically significant (*P* < 0.05).

RETRACTED

#### 4.2.3. Detection Results of Noncalcified Nodules

Here we use artificial intelligence software and radiologists to detect noncalcified nodules and analyze the size of the detected noncalcified nodules. The results are shown in Table 5.

It can be seen from Table 5 and Figure 3 that there are finally 236 true nodules, including 105 true nodules <5 mm, 79 true nodules 5–10 mm, and 52 true nodules >10 mm. The artificial intelligence software detected a total of 103 true nodules <5 mm, with a sensitivity of 98.1% and a sensitivity of 100% for detecting true nodules of 5–10 mm and >10 mm; radiologists detected a total of 19 true nodules <5 mm nodules and sensitivity was 18.1%, 32 true nodules 5–10 mm were detected, the sensitivity was 40.5%, and 47 true nodules >10 mm were detected, and the sensitivity was 90.4%. This shows that the sensitivity of artificial intelligence software to detect the size of noncalcified nodules is significantly higher than that of radiologists, and the difference is statistically significant (*P* < 0.05).

Here we use artificial intelligence software and radiologists to detect noncalcified nodules and analyze the nature of the detected noncalcified nodules. The results are shown in Table 6.

From Table 6 and Figure 4, it can be seen that finally there are 236 real nodules, including 79 real nodules with ground glass density, 26 real partial solid nodules, and 131 real solid nodules. The artificial intelligence software detected 78 terrestrial glass density real nodules with a sensitivity of 98.7%, 128 hard real nodules with a sensitivity of 97.7%, and some hard real nodules with a sensitivity of 100%. In radiology, doctors detected 23 real terrestrial glass density nodules with a sensitivity of 29.1%, 25 partial solid nodules with a sensitivity of 96.2%, and 43 solid real nodules with a sensitivity of 32.8%. This shows that the sensitivity of artificial intelligence software to detect the characteristics of uncalcified nodules is significantly higher than that of radiologists and that the difference is statistically significant (*P* < 0.05).

Here we use artificial intelligence software and radiologists to detect noncalcified nodules and analyze the positions of the detected noncalcified nodules. The results are shown in Table 7.

It can be seen from Table 7 and Figure 5 that there are finally 236 true nodules, of which 46 are true nodules at the junction of the pleura, 135 are true nodules at the peripheral junction and the true nodules at the center. 48 nodules and 7 true nodules are located in the hilar area. The sensitivity of artificial intelligence software to detect noncalcified nodules in the pleural, peripheral, central, and hilar areas is higher than that of radiologists, which shows that the sensitivity of artificial intelligence software to detect the location of noncalcified nodules is significantly higher than radiologists, and the difference was statistically significant (*P* < 0.05).

RETRACTED

### 4.3. CT Manifestations of Pulmonary Nodules

It can be seen from Figure 6 that, by comparing and analyzing the results of manual circles by experts, the algorithm proposed in this paper can accurately detect lung nodules and effectively eliminate the blood vessel endpoints and blood vessel intersection areas that cause false positives. The result is very close to the result manually delineated by the expert. Although the detection specificity needs to be further improved compared with the neural network classifier, the sensitivity is better than that of the neural network classifier, and the real-time performance is stronger. Since the task of the lung detection system is to assist the radiologist in diagnosis, the radiologist needs to make the final confirmation on the nodules automatically detected by the algorithm. Therefore, the algorithm focuses more on the sensitivity and real-time detection.

## 5. Conclusions

In this paper, based on a systematic analysis of domestic and international studies supporting the detection of pulmonary nodules in chest images, classification of pulmonary nodules in X-ray chest radiographs, detection and segmentation of rib markers, and detection and classification of pulmonary nodules in CT are done. In order to better classify the extracted suspect lung nodules, a pyramid feature network based on multiscale information is used to make the most of the multiscale spatial information to obtain better classification results. In this experiment, deep learning-based pulmonary nodule detection software is more sensitive than radiologists and can be used by doctors as an auxiliary detection tool to screen pulmonary nodules. Excluding nodules smaller than 5 mm reduces the false positive rate of the detection software. This article does not determine whether the detected pulmonary nodule is a benign or malignant pulmonary nodule, by looking for the entire process of detecting pulmonary nodules, that is, only the location of the pulmonary nodules. When a qualitative judgment is made about the lung nodules found, a radiologist can help diagnose the lung disease.

RETRACTED

## Figures and Tables

**Figure 1:** Indicator reliability test analysis chart.

**Figure 2:** Nodule detection sensitivity analysis chart.

**Figure 3:** Analysis of the results of noncalcified nodule size detection.

**Figure 4:** Analysis of the detection results of the properties of noncalcified nodules.

**Figure 5:** Analysis of the detection results of noncalcified nodules.

**Figure 6:** Analysis of CT findings of pulmonary nodules (https://image.baidu.com/). (a) Test results. (b) Experts manually circle the results.

**Table 1:** Data sheet of basic characteristics of patient nodules.

	Number of cases	Nodule type			Pathological type		Diameter		
		Ground glass density	Partial reality	Reality	Benign	Malignant	0-5 mm	5–10 mm	10–30 mm
Male	46	16	17	13	32	14	15	20	11
Female	34	9	14	11	27	7	11	15	8

**Table 2:** Data sheet of the evaluation index system for index reliability testing.

	Very clear	Clear	General	Not clear	Chaotic	Alpha
Pathological type	3.78	4.06	3.91	0.44	0.10	0.8192
Results of detection of noncalcified nodules	3.81	4.1	4.14	0.61	0.27	0.8536
Detection sensitivity	3.63	3.32	3.81	0.44	0.55	0.8273
False negative rate	3.63	3.74	4.44	0.38	0.19	0.7319
False positive rate	3.67	3.83	3.80	0.66	0.19	0.7267
CT findings of pulmonary nodules	3.87	3.92	4.62	0.34	0.23	0.8469

**Table 3:** Pathological type detection result data table.

	Benign	Malignant	Overall	Sensitivity (%)
Artificial intelligence software	59	21	80	100
Radiologist	59	21	80	100
Chest imaging expert + intelligent software	59	21	80	100

**Table 4:** Pathological type detection result data table.

	True nodule	False positive rate	≥5 mm false positive rate	Sensitivity (%)
Artificial intelligence software	234	2.4	1.2	99.15
Radiologist	112	0.02	0.01	47.45
Chest imaging expert + intelligent software	236	0	0	100

**Table 5:** Noncalcified nodule size detection result data table.

True nodule size (mm)	True nodule	Artificial intelligence software		Radiologist		*P*
		Number	Rate (%)	Number	Rate (%)	
<5	105	103	98.1	19	18.1	0.001
5–10	79	79	100	32	40.5	0.001
>10	52	52	100	47	90.4	0.005

**Table 6:** Noncalcified nodule nature detection result data table.

True nodule nature	True nodule	Artificial intelligence software		Radiologist		*P*
		Number	Rate (%)	Number	Rate (%)	
Reality	131	128	97.7	43	32.8	0.008
Partial reality	26	26	100	25	96.2	0.001
Ground glass	79	78	98.7	23	29.1	0.013

**Table 7:** Noncalcified nodule position detection result data sheet.

True nodule position	True nodule	Artificial intelligence software		Radiologist		*P*
		Number	Rate (%)	Number	Rate (%)	
Pleura connected	46	45	97.8	23	50.0	0.010
Peripheral	135	134	99.2	57	42.2	0.017
Centrality	48	47	97.9	21	43.8	0.004
Hilar area	7	7	100	3	42.9	0.042

RETRACTED

## Data Availability

No data were used to support this study.
